RETRACTED

# The Effectiveness Comparison of Different Acupuncture-Related Therapies on Knee Osteoarthritis: A Meta-Analysis

**DOI:** 10.1155/2022/2831332

**Published:** 2022-06-30

**Authors:** Chun Ye, Jianlong Zhou, Miaofen Wang, Shasha Xiao, Aihua Lv, Dejin Wang

**Affiliations:** ^1^Department of Emergency, Ningbo Traditional Chinese Medicine Hospital, Ningbo, Zhejiang Province 315010, China; ^2^Hand and Foot Trauma Surgery, Ningbo Ninth Hospital, Ningbo, Zhejiang Province 315032, China; ^3^Department of Traditional Chinese Medicine, Community Health Service Center, Baihe Street, Yinzhou District, Ningbo City, Zhejiang Province 315153, China; ^4^Department of Acupuncture and Moxibustion, Ningbo Medical Centre Lihuili Hospital, Ningbo University, Ningbo, Zhejiang 315040, China

## Abstract

**Objective:**

This meta-analysis aims to assess the efficacy of acupuncture-related therapy on knee osteoarthritis (KOA) patients.

**Method:**

We searched PubMed, Embase, and CNKI databases to screen eligible trials between 2017 and 2022. All trials that used acupuncture/moxibustion of KOA patients were included. Study selection and data extraction were performed by 2 researchers independently. The statistics was performed by using R 4.1.1.

**Results:**

A total of 17 trials were included in our meta-analysis. Meta-analysis results showed the evidence of the relation of several common acupunture/moxibustion treatments by network meta-analysis. In the fixed effect model, acupuncture/moxibustion has superior therapy efficacy than sham treatment (mean difference = −0.34, 95% confidence interval = (−0.52,−0.16), *P*=0.95). In fixed effect model, specific acupuncture/moxibustion has superior therapy efficacy than usual acupuncture/moxibustion (mean difference = –0.45, 95% confidence interval = (−0.62, −0.29), *P* < 0.01).

**Conclusion:**

Acupuncture/moxibustion has superior therapy efficacy than sham treatment. Specific acupuncture/moxibustion has superior therapy efficacy than usual acupuncture/moxibustion.

## 1. Introduction

Osteoarthritis (OA) is the most frequent reason for activity limitation in adults and is the most common type of arthritis [1, 2]. OA affects more than 240 million people in the world [1]. Patients with OA have more comorbidities than those without OA. Common management exercises, weight loss, education, and oral nonsteroidal anti-inflammatory drugs for patients without contraindications is given [3, 4]. Knee osteoarthritis (KOA) is the most common type of OA clinically [4–6]. Acupuncture and moxibustion are frequent traditional treatments for Chinese KOA patients.

Acupuncture and moxibustion are two traditional medical treatments in Chinese for thousands of years [7, 8]. Clinically, acupuncture and moxibustion are frequently used to apply to KOA [9, 10]. However, the effectiveness of acupuncture on KOA is still controversial. Acupuncture is considered to have little or no effect in reducing pain compared with sham treatment [4]. The evidence of the effectiveness of acupuncture on OA is limited and conflicting. We conduct this meta-analysis to investigate the therapeutic efficacy of acupuncture/moxibustion of KOA.

RETRACTED

## 2. Method

### 2.1. Literature Search

We searched PubMed, Embase, and CNKI to identify trials published from 2017 to 2022.

We searched PubMed with worlds “*osteoarthritis Acupuncture*” in all fields and limit to “*Clinical trial*” and “*Randomized Controlled Trial*” from 2017 to 2022.

We searched Embase PICO with the following strategy that “osteoarthritis”/exp AND “acupuncture”/exp AND “clinical trial”/exp AND [2017–2022]/py.

We searched CNKI with the following strategy in Chinese that *osteoarthritis Acupuncture* in *theme*. (Subject: Knee Arthritis (Precise)) AND (Subject: Acupuncture or Moxibustion (Precise)).

### 2.2. Inclusion Criteria

We included patients with KOA. Studies conducted interventions that moxibustion and acupuncture were included in our study. Acupuncture that electroacupuncture, manual acupuncture, and some other specific acupunctures were included. The intervention duration was usually 4 weeks or 8 weeks.

### 2.3. Exclusion Criteria

The intervention of literature that included pharma, rehabilitation, or excise was excluded from our study. Literature review, case report, or protocols were excluded.

### 2.4. Outcomes and Data Extraction

The primary outcome was the response rate after interventions. The secondary outcome was the Western Ontario and McMaster Universities Osteoarthritis Index (WOMAC) function scale. The two outcomes were extracted from the original literature. Two researchers conducted literature selection individually.

### 2.5. Statistical Analysis

We performed network meta-analyses to compare data from individual trials. Fixed effects meta-analyses were used to incorporate data from individual trials separately. Effects on continuous outcomes were measured by mean differences (MDs). Sensitivity analyses were performed to test the robustness of the estimates so that the exclusion of studies was with a high overall risk of bias. The *gemtc*, *rjags*, and *meta* package in R version 4.1.1 were used for the statistic and plotting.

## 3. Results

### 3.1. Study Screening

We found 462 papers in PubMed, Embase, and CNKI. After literature selection, we finally selected 17 papers for our study (Figure 1). All of the 17 studies reported the primary outcome and 10 of them report the WOMAC function score. The control arm was sham acupuncture or sham moxibustion in 5 of the 17 studies. The control arm was acupuncture in 6 of the 17 studies (Table 1).

RETRACTED

### 3.2. Network of the Response Rate

In all selected 17 literature, the relationship between acupuncture and electroacupuncture and the relationship between acupuncture and moxibustion show stronger evidence than other acupuncture-related treatments (Figure 2).

### 3.3. Comparison between Acupuncture/Moxibustion and Sham Treatment

5 studies reported WOMAC functional scores. When a paper published by Zhao 2021 [20] is included, *I*^2^ = 95% (Figure 3(a)). We next did sensitivity analysis of these 5 literature. Also, the paper by Zhao et al. [20] showed a high overall risk of bias (Figure 3(b)). So, we excluded the paper by Zhao et al. [20] and analyzed it again (Figure 3(c)). As shown in Figure 3(c), in the fixed effect model, acupuncture/moxibustion had a superior therapy effect than sham treatment.

### 3.4. Comparison between Specific Acupuncture and Usual Acupuncture

We compared specific acupuncture/moxibustion vs. usual acupuncture in the fixed effect model. As shown in Figure 4(a), specific acupuncture/moxibustion had a superior therapy effect than usual acupuncture. Also, the sensitivity analysis of the 6 papers was not shown a risk of bias (Figure 4(b)).

### 3.5. Publish Bias

A significant publication bias was found for both the comparison of acupuncture/moxibustion vs. sham treatment and the comparison of specific acupuncture/moxibustion vs. usual acupuncture (Figures 5(a) and 5(b)).

## 4. Discussion

The meta-analysis included 17 trials to assess the efficacy of acupuncture/moxibustion in treating KOA. Network analysis of the comparison between acupuncture/moxibustion, sham treatment, or specific acupuncture/moxibustion shows that evidence mainly among the relation between acupuncture, electroacupuncture, and moxibustion in KOA patients (Figure 2). Meta-analysis of comparison between acupuncture/moxibustion vs. sham treatment shows that acupuncture/moxibustion has superior therapy efficacy to sham treatment in KOA patients on WOMAC function (Figure 3). Meta-analysis of comparison between specific acupuncture/moxibustion has superior therapy efficacy than usual acupuncture in KOA patients on WOMAC function (Figure 4). Herein, the effects of acupuncture and moxibustion therapy on the WOMAC function scale were investigated. We compare the WOMAC function score for most studies that have reported it. Moreover, electroacupuncture was superior to sham treatment.

In Liu et al.'s study, the result of a network meta-analysis was to draw a familiar conclusion to our analysis [26]. Similar to our result, moxibustion is effective and the level of evidence is moderate in Choi et al.'s paper [27]. A meta-analysis of previous online studies on the subject found that warm needle and electroacupuncture were probably the best acupuncture modalities for treating KOA [28]. Lots of papers report the efficacy of acupuncture [26, 28, 29]. However, few of them have firm foundation data. That is why the efficacy of acupuncture and moxibustion is contradictory in the world.

RETRACTED

Because acupuncture and moxibustion are traditional therapy in China and most of the literature has come from China, there is an unavoidable publish bias that existed. The low quality of the selected literature may lead to adventurous conclusions, which should be carefully analyzed.

In conclusion, our meta-analysis indicated that acupuncture/moxibustion has superior therapeutic efficacy than sham treatment. Also, specific acupuncture/moxibustion has superior therapy efficacy than usual acupuncture/moxibustion.

## Figures and Tables

**Figure 1:** Flowchart of study screening.

**Figure 2:** Network of the response rate of the selected papers. A: acupuncture; B: electroacupuncture; C: sham; D: moxibustion; E: special acupuncture; F: special moxibustion.

**Figure 3:** Analysis of comparison between acupuncture/moxibustion vs. sham treatment. (a) Forest plot of data included in the study by Zhao et al. [20]. (b). Sensitivity analysis of data included in the study by Zhao et al. [20]. (c). Forest plot of data without the study by Zhao et al. [20].

**Figure 4:** Analysis of comparison between specific acupuncture/moxibustion vs. usual acupuncture. (a) Forest plot of specific acupuncture/moxibustion vs. usual acupuncture. (b) Sensitivity analysis of the 6 literature.

**Figure 5:** Funnel plot of the papers reported WOMAC. (a) Funnel plot of comparison of acupuncture/moxibustion and sham treatment. (b) Funnel plot of comparison of specific acupuncture/moxibustion and usual acupuncture.

**Table 1:** Patients' characteristic of the included studies.

Author	year	Experiment	Fluquency	Duration time	e.N	e.WOMAC function score	Control	con.N	con.WOMAC function score
Ton et al. [11]	2021	Acupuncture	—	—	120	—	No acupuncture	179	—
Wang et al. [12]	2020	Electroacupuncture	—	8w	15	—	Sham electroacupuncture	15	—
Chen et al. [13]	2020	Electroacupuncture	—	—	28	—	Acupuncture	28	—
Liang et al. [14]	2019	Soft-tissue relaxing needing	1 time/2 d	4times	20	—	Electroacupuncture	20	—
Chen et al. [15]	2018	Acupuncture	—	—	30	—	-	—	—
Chen et al. [15]	2018	Aconite cake-separated moxibustion	—	—	30	—	Moxibustion	30	—
Deng et al. [16]	2020	Stuck-needle technique	—	—	33	—	Regular acupuncture	32	—
Wang et al. [17]	2017	Warm needling moxibustion	—	—	25	11.0 ± 8.99	Sham	21	15.86 ± 11.30
Wang et al. [18]	2020	Electroacupuncture	—	8 W	43	11.39 ± 7.34	Acupuncture	30	14.86 ± 8.06
Shi et al. [19]	2020	Electroacupuncture	—	8 w	28	11.39 ± 7.34	Manual acupuncture	30	14.86 ± 8.06
Zhao et al. [20]	2021	Laser moxibustion	—	4 w	193	11.69 ± 14.19	Sham laser control group	177	1.38 ± 6.35
Lin et al. [21]	2020	Intensive acupuncture	3 sessions/w vs.1 session/w	8 w	30	14.5 ± 8.3	Acupuncture	30	17.5 ± 6.9
Chen et al. [22]	2020	Moxibustion	—	4 w	28	14.86 ± 4.03	Acupuncture	28	23.75 ± 6.88
Yu W	2021	Acupuncture	—	—	61	27.89 ± 16.85	Sham acupuncture	31	32.58 ± 18.58
Fu et al. [23]	2021	Fire needling	—	2 w	26	7.92 ± 3.89	Regular acupuncture	26	11.58 ± 7.60
Tu et al. [24]	2021	Electro-acupuncture	3 times/w	8 w	151	9.26 ± 7.03	Sham acupuncture	146	11.78 ± 8.17
Fu et al. [25]	2020	Miao crossbow needle	normal, 3 times/w, 20 w	46 d	149	9.35 ± 6.73	Acupuncture	152	11.41 ± 7.49

RETRACTED

## Data Availability

The data can be obtained from the author upon reasonable request.
